The article "Antimicrobial Step-Down Therapy versus Conventional Antimicrobial Therapy in the Treatment of Patients with Sepsis" was retracted in 2023. Reasons: suspected computer-generated content; unreliable results or conclusions; concerns about the data; concerns about the results or conclusions.

# Antimicrobial Step-Down Therapy versus Conventional Antimicrobial Therapy in the Treatment of Patients with Sepsis

**DOI:** 10.1155/2022/3117805

**Published:** 2022-08-31

**Authors:** Zhuo Peng, Zequn Niu, Rui Zhang, Longfei Pan, Hui Feng, Yang Zhou, Honghong Pei

**Affiliations:** Emergency Department, The Second Affiliated Hospital of Xi'an Jiaotong University, Xi'an, Shaanxi Province 710000, China

## Abstract

**Objective:**

This study was to evaluate the efficacy of antimicrobial step-down therapy versus conventional antimicrobial therapy in the treatment of patients with sepsis.

**Methods:**

Between September 2020 and September 2021, 65 patients with sepsis treated in the intensive care unit (ICU) of our hospital were recruited and assigned at a ratio of 1 : 1 to receive either conventional antimicrobial therapy (sulbactam plus cefoperazone) (control group) or antimicrobial step-down therapy (imipenem/cilastatin) (observation group). The results of drug sensitivity tests and clinical effects were evaluated comprehensively after 3-5 d of treatment, downgraded, and upgraded, or maintenance treatment was administered for 10 d. Outcome measures included clinical and laboratory indices and treatment efficacy.

**Results:**

Antimicrobial step-down therapy resulted in a significantly higher efficacy and lower levels of white blood cell (WBC) count and C-reactive protein (CRP) versus conventional antimicrobial therapy (*P* < 0.05). The patients given antimicrobial step-down therapy showed a significantly shorter duration of antimicrobial drug administration, temperature recovery, time of respiratory support, and ICU stays versus conventional antimicrobial therapy (*P* < 0.05).

**Conclusion:**

Antimicrobial step-down therapy contributes to the mitigation of inflammatory responses in patients with sepsis and shortens the duration of antimicrobial drug use and ICU stay versus conventional antimicrobial therapy. The reliability of the conclusions can be further increased if multicenter and large sample clinical observations can be conducted, which is the direction of endeavor for future clinical studies.

## 1. Introduction

Sepsis is a life-threatening organ dysfunction caused by a dysregulated host response to infection and is one of the leading causes of death in children. Early use of antimicrobial drugs can improve prognosis, and the 2020 international guidelines recommend the empirical use of broad-spectrum antimicrobial drugs to cover all possible pathogenic microorganisms. However, overuse of broad-spectrum antimicrobial drugs is associated with the development of bacterial resistance.

Anti-infection treatment is one of the key approaches to lower the morbidity and mortality rate and improve the quality of survival in patients with sepsis [1]. Traditional anti-infective treatment is mostly empirical, which is predisposed to antibiotic abuse, drug resistance, and compromised therapeutic efficiency [2, 3]. According to international recommendations for severe sepsis and septic shock management, antimicrobial medication step-down therapy may serve as a reference strategy for the first anti-infective treatment of sepsis patients [4]. Moreover, a growing body of evidence has confirmed that the above-mentioned anti-infective treatment could effectively relieve the clinical symptoms of patients with acute and critical infections [5, 6] and prevent the adverse events associated with repeated changes of antimicrobial drugs due to drug resistance [7]. In a 2015 epidemiological survey, the mortality rate of sepsis in the ICU was 36% in China and 24%-40% in Europe. Thus, it is of great importance to find appropriate drug treatment to improve the prognosis. In traditional Chinese medicine (TCM), sepsis belongs to the categories of “warm poison” and “typhoid fever,” while severe septic shock belongs to the category of “derangement” and “mental fainting.” Multiorgan dysfunction syndrome is reflected in the malfunction of the five organs.

The article "Antimicrobial Step-Down Therapy versus Conventional Antimicrobial Therapy in the Treatment of Patients with Sepsis" was retracted in 2023. Reasons: suspected computer-generated content; unreliable results or conclusions; concerns about the data; concerns about the results or conclusions.

With the rapid development of social science and medical technology, a series of new therapeutic protocols and strategies have been adopted for treatment based on pharmacological theories and the effects and practical implications. Antimicrobial step-down therapy is a summary of empirical treatment plan for anti-infection, which is also one of the strategies for optimal antimicrobial drug treatment applied in China at present. It provides unique advantages in clinical anti-infection treatment.

In this prospective study, 65 patients with sepsis were recruited between September 2020 and September 2021 to evaluate the efficacy of antimicrobial step-down therapy in patients with sepsis and to provide a more theoretical basis for clinical practice.

## 2. Materials and Methods

### 2.1. Baseline Data

Between September 2020 and September 2021, 65 patients with sepsis treated in the intensive care unit (ICU) of our hospital were recruited and assigned at a ratio of 1 : 1 to receive either conventional antimicrobial therapy (control group, *n* = 31) or antimicrobial step-down therapy (observation group, *n* = 34).

The randomization was carried out using an online web-based randomization tool (freely available at http://www.randomizer.org/). For concealment of allocation, the randomization procedure and assignment were managed by an independent research assistant who was not involved in screening or evaluation of the participants.

The article "Antimicrobial Step-Down Therapy versus Conventional Antimicrobial Therapy in the Treatment of Patients with Sepsis" was retracted in 2023. Reasons: suspected computer-generated content; unreliable results or conclusions; concerns about the data; concerns about the results or conclusions.

The original sample size calculation estimated that 100 patients in each group would be needed to detect a 3-point difference between groups in a 2-sided significance test with a power of 0.8 and an alpha error level of 0.05.

The trial was done in accordance with standards of Good Clinical Practice and the Declaration of Helsinki. The trial protocol and all amendments were approved by the appropriate ethics body at each participating institution. All patients provided written informed consent before enrolment. The trial protocol has been published online and is available with the full text of this article. Ethics number: LI-LO20200908.

In the observation group, there were 21 males and 13 females, aged 36-75 (58.98 ± 6.42) years. In the control group, there were 19 males, and 12 females, aged 38-78 (59.11 ± 6.53) years. Patients and their families were fully informed of the process of the study and provided written informed consent.

Inclusion criteria: ① aged 18 to 80 years; ② met the relevant diagnostic criteria for sepsis [8]; ③ with an expected survival of ≥3 d.

Exclusion criteria: ① with antimicrobial therapy before enrollment; ② with mixed or fungal infections; ③ with liver, kidney, and heart failure; ④ with malignant tumors and immune system diseases; ⑤ with the use of hormones or immunosuppressive drugs within the last 3 months; ⑥ with a history of allergy to the drug; ⑦ subjects or their family members who do not cooperate with the enrollment group for treatment; ⑧ those with incomplete medical history; ⑨ those who have participated in other clinical trials.

### 2.2. Treatment Methods

Both groups of patients received conventional treatment such as nutritional support, organ function support, respiratory support (oxygen or mechanical ventilation), fluid replacement, blood pressure, and blood glucose control after admission to ICU. The control group received 2.0 g of sulbactam and cefoperazone (Beijing Taiyang Pharmaceutical Co., Ltd., GMP H20045208) by intravenous infusion with an interval of 8 h between doses. After 3-5 d of treatment, the results of the drug sensitivity test and clinical effect were comprehensively evaluated, followed by downgraded, upgraded, or maintenance treatment for 10 d. The observation group received 1.0 g of imipenem/cilastatin (Haisheng Pfizer Pharmaceutical Co., Ltd., State Pharmacopoeia H20067765, specification 1.0 g) by intravenous infusion with an interval of 8 h between doses. After 3-5 d of treatment, the results of the drug sensitivity test and clinical effect were comprehensively evaluated, downgraded, and upgraded, or maintenance treatment was administered for 10 d.

The article "Antimicrobial Step-Down Therapy versus Conventional Antimicrobial Therapy in the Treatment of Patients with Sepsis" was retracted in 2023. Reasons: suspected computer-generated content; unreliable results or conclusions; concerns about the data; concerns about the results or conclusions.

The two groups received Banxia Xiexin decoction. Pinelliae Rhizoma 9 g, Scutellariae Radix 9 g, Coptidis Rhizoma 6 g, ginseng 9 g, dried ginger 9 g, roasted liquorice root 9 g, and 4 jujubes were decocted with water to obtain 100 mL of filtrate and administered nasally in the morning and evening with an interval of 12 h. The herbs were decocted by the decoction room of Shandong Provincial Hospital. The duration of treatment was 1 week.

### 2.3. Outcome Measures

#### 2.3.1. Laboratory Indicators

Venous blood was collected from patients before and after treatment, and white blood cell (WBC) and C reactive protein (CRP) levels were determined with a fully automated biochemical analyzer from Beckman Coulter (Model AU680), USA.

#### 2.3.2. Clinical Indices

The duration of temperature recovery, the time of respiratory support, and the time of ICU stay were recorded in both groups. Body temperature was measured using a mercury thermometer to determine axillary temperature, with a normal body temperature of 37.3°C. The height and weight of the patients were measured on admission to the ICU, the body mass index (BMI) was calculated, and the Acute Physiology and Chronic Health Evaluation II (APACHE II) system were used to assess the patients' condition.

#### 2.3.3. Clinical Efficacy

Markedly effective: after treatment, the patients' clinical indexes and laboratory indexes returned to normal and clinical signs disappeared. Effective: after treatment, clinical and laboratory indices were improved, and clinical signs disappeared. Ineffective: after treatment, no improvement or worsening of clinical indices, laboratory indices, or clinical signs was observed.

(1) $$\begin{array}{c} \text{Efficacy}=\frac{\left(\text{markedly effective cases}+\text{effective cases}\right)}{\text{total number of cases}}*100\%. \end{array}$$

### 2.4. Statistical Analysis

If the parameter beta is either a difference of means, a log odds ratio, or a log hazard ratio, then it is reasonable to assume that *b* is unbiased and normally distributed.

SPSS 20.0 was used for data analyses. The measurement data were expressed as ($\bar{x}\pm s$) and processed using the independent sample *t*-test. The count data were expressed as the number of cases (rate) and analyzed using the chi-square test. Differences were considered statistically significant at *P* < 0.05.

## 3. Results

### 3.1. Patient Characteristics

There were no statistically significant differences in age, BMI, body temperature, heart rate, APACHE II score, type of primary disease, and blood pathogenic bacteria species between the two groups (*P* > 0.05) (Table 1).

### 3.2. Clinical Efficacy

Antimicrobial step-down therapy was associated with a significantly higher efficacy versus conventional antimicrobial therapy (*P* < 0.05). (Table 2).

The article "Antimicrobial Step-Down Therapy versus Conventional Antimicrobial Therapy in the Treatment of Patients with Sepsis" was retracted in 2023. Reasons: suspected computer-generated content; unreliable results or conclusions; concerns about the data; concerns about the results or conclusions.

### 3.3. Laboratory Indices

Antimicrobial step-down therapy resulted in significantly lower levels of WBC count and CRP versus conventional antimicrobial therapy (*P* < 0.05). (Table 3).

### 3.4. Clinical Indices

Patients who received antimicrobial step-down therapy required shorter antimicrobial medication administration, temperature recovery, respiratory support, and ICU stays than those who received traditional antimicrobial therapy (*P* < 0.05) (Table 4).

## 4. Discussion

Sepsis is an important disease in the field of acute and critical care, which may be complicated by multiorgan dysfunction and septic shock, with an annual prevalence of approximately 19 million worldwide, and a mortality rate of between 24% and 40% in European countries and 20% in the United States [9]. In a comprehensive ICU epidemiological survey of major tertiary hospitals in China in 2015, the sepsis morbidity and mortality rate was 36%. Patients with sepsis frequently suffer from organ dysfunction caused by infection, leading to organ failure until death [10]. In addition to aggressive treatment of the primary disease and supportive therapy, anti-infective therapy is an important part in sepsis management [11, 12]. A recent study on bacterial pathogenesis and antimicrobial resistance in sepsis patients in ICU found that patients with sepsis had a wide variety of bacterial infections, including *S. aureus* and *Escherichia coli* with high resistance, and the results suggested the significance of a rational selection and use of antibiotics [13, 14].

Previously, conventional antimicrobial therapy adopted an ascending stepwise model, which has been shown to be effective in patients with mild infections. However, for severe infection cases, despite certain mitigation on the APACHE II score and inflammatory response [15], it is mostly substituted by cephalosporins with higher potency due to its suboptimal efficacy, which increases the risk of adverse effects and the development of drug-resistant bacteria [16]. As a result, “step-down treatment” was recommended as a sensible medication approach for antimicrobial drug usage in ICU patients with severe bacterial infections. A step-down regimen used in the clinical treatment of elderly patients with severe pneumonia in the ICU has been proven to be highly effective, improving all blood gas indicators and decreasing the period of symptom alleviation and hospitalization [17].

In the present study, the results showed that antimicrobial step-down therapy was associated with a significantly higher efficacy (85.29%) versus conventional antimicrobial therapy (61.29%), which was consistent with previous research results [18, 19]. The efficacy of the convention antimicrobial therapy was lower than the results of prior research [20], which may be attributed to the limited number of study participants. The results indicate that the antimicrobial step-down therapy features a promising clinical efficacy. Step-down therapy is an empirical anti-infective regimen with the following two characteristics: (1) a single, broad-spectrum, potent antibiotic is used at the beginning of anti-infective therapy to cover as many germs as possible that may cause the infection; (2) after 48-72 h, the antibiotics are adjusted according to the results of microbiological examination of drug sensitivity to be more targeted. It is a new treatment strategy adopted in recent years for severe bacterial infections [21, 22]. The strategy consists of two phases: the first phase is empirical treatment with broad-spectrum antibiotics, and the second phase is downgrading to a relatively narrow spectrum of antibiotics, which is the adjustment of relatively narrow-spectrum, targeted antibiotic species according to microbiological examination and drug sensitivity results, to shorten the course of treatment, and to maximize the best possible efficacy of anti-infective treatment [23]. The aim is to increase survival, improve patient prognosis, reduce bacterial resistance, avoid the adverse effects of broad-spectrum antibiotics, and balance the differences in needs between individual patients and society. The two phases of “empirical treatment” and “targeted treatment” are unified and organically combined to form an integrated step-down treatment program [24].

The article "Antimicrobial Step-Down Therapy versus Conventional Antimicrobial Therapy in the Treatment of Patients with Sepsis" was retracted in 2023. Reasons: suspected computer-generated content; unreliable results or conclusions; concerns about the data; concerns about the results or conclusions.

Moreover, antimicrobial step-down therapy resulted in significantly lower levels of WBC count and CRP versus conventional antimicrobial therapy, indicating that antimicrobial step-down therapy facilitates the alleviation of inflammatory responses in the patients. In addition, the patients given antimicrobial step-down therapy showed a significantly shorter duration of antimicrobial drug administration, time of temperature recovery, time of respiratory support, and ICU stays versus conventional antimicrobial therapy, suggesting the value of step-down antimicrobial therapy in the anti-infective treatment of patients with sepsis, which can effectively improve patients' prognosis and reduce their psychological and economic burden.

TCM treatment for sepsis mainly includes the internal treatment methods of clearing heat and detoxification, activating blood circulation and eliminating blood stasis, supporting the root, and attacking the lower and inner parts of the body. The external treatment method includes enema method, acupuncture and moxibustion, and acupuncture point compressing. Banxia Xiexin decoction [25] is preferred for the treatment of sepsis by regulating the qi. Banxia Xiexin decoction regulates spleen and stomach qi, improves organ function, and reduces the occurrence of gastrointestinal abscesses, perforations, and adhesions through various mechanisms such as improving intestinal permeability, reducing inflammatory response, inhibiting vascular permeability, and reducing neutrophil aggregation. Scutellariae Radix glycosides, berberine hydrochloride, and complexes of Scutellariae Radix glycosides and berberine in the formula have antibacterial activity, regulate the imbalance of intestinal microecology, improve the absorption of nutrients in the gastrointestinal tract, and ensure the energy intake of the body and the regulation of inflammatory response [26, 27].

The article "Antimicrobial Step-Down Therapy versus Conventional Antimicrobial Therapy in the Treatment of Patients with Sepsis" was retracted in 2023. Reasons: suspected computer-generated content; unreliable results or conclusions; concerns about the data; concerns about the results or conclusions.

At present, clinicians in large- and medium-sized urban hospitals, especially ICU clinicians, have a full understanding of step-down therapy and can timely retain pathogen culture specimens, with the rational use of antibacterial drugs. However, a significant proportion of clinicians have insufficient knowledge of step-down therapy, resulting in increased morbidity and mortality, drug resistance, or drug costs. Therefore, clinical academic exchanges among medical institutions at all levels should be strengthened to raise awareness of the use of step-down therapy as an empirical anti-infective treatment option for patients with acute and critical infections.

To sum up, antimicrobial step-down therapy contributes to the mitigation of inflammatory responses in patients with sepsis and shortens the duration of antimicrobial drug use and ICU stay versus conventional antimicrobial therapy. Multicenter and large sample clinical observations will be conducted in the future to further increase the reliability of the findings. The clinical efficacy and safety of Chinese medicine combined with antibacterial drug step-down therapy for sepsis is gradually gaining extensive acceptance, and the treatment strategy of combining Chinese and Western medicine is expected to be better promoted.

## Figures and Tables

**Table 1:** Comparison of baseline data.

Items	Observation group (*n* = 34)	Control group (*n* = 31)	*t*/*χ*^2^	*P* value
Age (year, _cc_)	58.98 ± 6.42	59.11 ± 6.53	0.081	0.936
BMI (kg/m^2^, $\bar{x}\pm s$)	19.21 ± 2.54	19.34 ± 2.63	0.203	0.840
Body temperature (°C, $\bar{x}\pm s$)	38.47 ± 0.58	38.51 ± 0.62	0.269	0.789
Heart rate (time/min, $\bar{x}\pm s$)	114.59 ± 16.89	114.63 ± 16.71	0.010	0.992
APACHEII (points, $\bar{x}\pm s$)	26.12 ± 4.78	25.93 ± 4.81	0.160	0.874
Primary disease			2.438	0.743
Severe multiple injuries	11	9		
Severe pneumonia	5	7		
Acute severe pancreatitis	8	8		
Acute severe cholangitis	9	6		
Postoperative secondary infection	1	1		
Blood-borne pathogens			1.145	0.285
Gram-negative bacteria	21	23		
Gram-positive bacteria	13	8		

The article "Antimicrobial Step-Down Therapy versus Conventional Antimicrobial Therapy in the Treatment of Patients with Sepsis" was retracted in 2023. Reasons: suspected computer-generated content; unreliable results or conclusions; concerns about the data; concerns about the results or conclusions.

**Table 2:** Comparison of clinical efficacy [*n* (%)].

Groups	*n*	Markedly effective	Effective	Ineffective	Efficacy
Observation group	34	22	7	5	29/85.29
Control group	31	13	6	12	19/61.29
*χ* ^2^					4.838
*P* value					0.028

**Table 3:** Comparison of laboratory indices ($\bar{x}\pm s$).

Groups	*n*	WBC (×10^9^/L)		CRP (mg/L)	
		Before treatment	After treatment	Before treatment	After treatment
Observation group	34	17.89 ± 1.45	6.11 ± 1.34^a^	91.25 ± 12.36	20.15 ± 5.37^a^
Control group	31	17.76 ± 1.48	9.78 ± 1.31^a^	89.57 ± 12.44	39.48 ± 5.43^a^
*t* value		0.357	11.147	0.546	14.418
*P* value		0.722	0.001	0.587	0.001

Note: ^a^ indicates a significant difference (*P* < 0.05) in the comparison with before treatment.

**Table 4:** Comparison of clinical indices ($\bar{x}\pm s$).

Groups	*n*	Time of antimicrobial drug administration (d)	Time of temperature recovery (d)	Time of respiratory support (d)	ICU stay (d)
Observation group	34	10.98 ± 1.67	4.11 ± 1.25	4.97 ± 2.11	14.65 ± 2.47
Control group	31	13.26 ± 1.64	5.34 ± 1.23	6.42 ± 1.98	18.28 ± 2.54
*t* value		5.545	3.993	2.849	5.839
*P* value		0.001	0.001	0.006	0.001

## Data Availability

All data generated or analyzed during this study are included in this published article.
